The article "The Diarylheptanoid Curcumin Induces MYC Inhibition and Cross-Links This Oncoprotein to the Coactivator TRRAP" was published in 2021. Journal: Front Oncol.

# The Diarylheptanoid Curcumin Induces MYC Inhibition and Cross-Links This Oncoprotein to the Coactivator TRRAP

**DOI:** 10.3389/fonc.2021.660481

**Published:** 2021-04-15

**Authors:** Alexander Mödlhammer, Sandra Pfurtscheller, Andreas Feichtner, Markus Hartl, Rainer Schneider

**Affiliations:** Institute of Biochemistry and Center for Molecular Biosciences Innsbruck (CMBI), University of Innsbruck, Innsbruck, Austria

**Keywords:** gene regulation, transcription control, cancer, protein modification, cell transformation

## Abstract

The c-Myc protein (MYC) is a transcription factor with strong oncogenic potential controlling fundamental cellular processes. In most human tumors, MYC is overexpressed by enhanced transcriptional activation, gene amplification, chromosomal rearrangements, or increased protein stabilization. To pharmacologically suppress oncogenic MYC functions, multiple approaches have been applied either to inhibit transcriptional activation of the endogenous *MYC* gene, or to interfere with biochemical functions of aberrantly activated MYC. Other critical points of attack are targeted protein modification, or destabilization leading to a non-functional MYC oncoprotein. It has been claimed that the natural compound curcumin representing the principal curcumoid of turmeric (*Curcuma longa*) has anticancer properties although its specificity, efficacy, and the underlying molecular mechanisms have been controversially discussed. Here, we have tested curcumin’s effect on MYC-dependent cell transformation and transcriptional activation, and found that this natural compound interferes with both of these MYC activities. Furthermore, in curcumin-treated cells, the endogenous 60-kDa MYC protein is covalently and specifically cross-linked to one of its transcriptional interaction partners, namely the 434-kDa transformation/transcription domain associated protein (TRRAP). Thereby, endogenous MYC levels are strongly reduced and cells stop to proliferate. TRRAP is a multidomain adaptor protein of the phosphoinositide 3-kinase-related kinases (PIKK) family and represents an important component of many histone acetyltransferase (HAT) complexes. TRRAP is important to mediate transcriptional activation executed by the MYC oncoprotein, but on the other hand TRRAP also negatively regulates protein stability of the tumor suppressor p53 (TP53). Curcumin-mediated covalent binding of MYC to TRRAP reduces the protein amounts of both interaction partners but does not downregulate TP53, so that the growth-arresting effect of wild type TP53 could prevail. Our results elucidate a molecular mechanism of curcumin action that specifically and irreversibly targets two crucial multifunctional cellular players. With regard to their broad impact in cancer, our findings contribute to explain the pleiotropic functions of curcumin, and suggest that this natural spice, or more bioavailable derivatives thereof, may constitute useful adjuvants in the therapy of MYC-dependent and TRRAP-associated human tumors.

## Introduction

The transcription factor MYC is a master regulator of fundamental cellular processes like growth and proliferation (1–3), and constitutes the central hub of a regulatory network controlling the expression of thousands of genes. Hyperactivation of *MYC* occurs in the majority of all human cancers classifying this protooncogene as a major cancer driver (3–8). MYC is a bHLH-LZ protein encompassing protein dimerization domains (helix-loop-helix, leucine zipper) and a DNA contact surface (basic region) that forms heterodimers with the MAX protein and typically binds to specific DNA sequence elements termed E‑boxes (2, 9). To fulfill its transcriptional regulatory tasks, MYC has to interact with multiple components of the transcriptional machinery *via* non-covalent associations (10). Among those interaction partners are cofactors like the 434-kDa coactivator TRRAP (transformation/transcription domain associated protein) recruiting histone H3 and H4 acetyltransferase activities (2, 11, 12). Thereby, TRRAP interacts with the MYC-Box II (MBII) and N-terminally adjacent to MYC-Box I (MBI), both binding sites located in the N-terminal transactivation domain of MYC. Besides TRRAP, other coactivators like EP400 (p400), GCN5, or TIP60 form MBII-dependent complexes for regulating MYC’s transcriptional functions (2, 13). In case of EP400, the interaction with MYC *via* TRRAP is relevant for the transforming activity of the human adenovirus 5 E1A protein (14, 15). Likewise, TRRAP is required for MYC-dependent cell transformation (16) but on the other hand TRRAP is also needed to maintain a tumor-suppressive high level of the wildtype TP53 protein in normal cells, as well as tumorigenesis-promoting high levels of mutated TP53 in cancer cells (17). In this context, TRRAP is essential for regulating TP53 accumulation in lymphoma and for transcriptional activation of *MDM2* encoding an E3-ubiquitin ligase. MDM2 marks wild type TP53 for proteasomal degradation within a negative feedback regulation loop keeping TP53 levels low in normal cells (17, 18). In addition, a putative tumor-suppressive role of TRRAP has been described in breast carcinomas where TRRAP is significantly downregulated compared to normal breast tissues, and lower TRRAP expression correlates with a shorter survival time (19).

The diarylheptanoid curcumin [(1E,6E)-1,7-Bis(4-hydroxy-3-methoxyphenyl)hepta-1,6-diene-3,5-dione] represents the principal curcumoid of turmeric (*Curcuma longa*). This polyphenolic pigment is generated in the root and normally used as a spice, or as approved food dye (E100), but is also in medicinal use since ancient times to treat diverse diseases such as rheumatism, fever, intestinal disorder, trauma, and amenorrhea (20). This wide therapeutic spectrum may be due to the pleiotropic effects of curcumin including anti-inflammatory, immunomodulatory, antimalarial, and anti-cancer properties (20). The natural yellow color of curcumin is caused by the phenol groups in the diarylheptanoid structure, which has a tautomeric character existing in an enolic and in a keto form. Due to its chemical structure, curcumin displays a high chemical reactivity with multiple biological targets. The 1,3-dicarbonyl group is a potential chelator for metal ions, the two α, β-unsaturated systems in the enolic moiety are potent Michael acceptors for sulfhydryl groups, and the two phenolic groups are susceptible to redox reactions (21). Due to its multiple reactivities, the compound displays poly-pharmacological effects as outlined above, which may be also mediated by the covalent adduction of curcumin to distinct cellular proteins through a Michael-type addition (21).

The curcumin-containing foodstuff turmeric is widely applied in traditional medicine and has been extensively tested for its therapeutic use. This resulted in the documentation of many unspecific effects classifying turmeric/curcumin as one of the so-called pan-assay interference compounds, or invalid metabolic panaceas (20, 22). Several clinical trials attest curcumin to be an unstable and reactive compound with poor bioavailability (23). However, other clinical studies have demonstrated specific efficacies pointing at least to some therapeutic benefits, which would justify further investigations on curcumin’s molecular targets and their regulatory mechanisms (24, 25). Besides its anti-inflammatory properties, there is mounting evidence from many pre-clinical and several clinical studies that curcumin also has anticancer properties by preventing tumorigenesis, dissemination, and metastasis in tumor cells (26–29). Thereby, curcumin leads to decreased mRNA-levels of *MYC*, insulin, and IGF-1 receptors, which could cause the observed anti-growth and anti-migration properties for instance in colorectal cancer cells (26). Therefore, curcumin as a nutraceutical could be useful in the prevention and adjuvant therapy for instance in colorectal neoplasia (20, 30, 31).

Here we show that curcumin inhibits MYC-induced cell transformation and transcriptional activation, and that this compound cross-links MYC with one of its direct interactors, namely the coactivator TRRAP. This leads to significantly lower free MYC but almost unchanged TP53 levels in the tested cells, which may be responsible for the observed growth arrest. Our results point to a novel molecular mechanism, which would allow to drug the multifaceted MYC oncoprotein by specifically cross-linking it covalently to a functionally crucial interaction partner. This mechanism is not only a new paradigm in drug-development but may pave the way to understand the principles underlying the multiple functions associated with the plant ingredient curcumin.

## Materials and Methods

### Cell Culture and Cell Transformation Assay

Primary quail embryo fibroblasts (QEF) were prepared from 9-d old fertilized quail eggs and cells cultivated as described (32). Calcium phosphate-mediated transfection of DNA into fibroblasts and quantification of cell transformation by focus formation were performed as described (33, 34). Cultivation and DNA transfection of human epithelial kidney cells (HEK‑293T) by lipofection have been described (35).

### Expression Plasmids, Gene Transfer, Reporter Gene Assay, and Cell Proliferation Analysis

The pRc/RSV-derived eukaryotic expression vectors pRc-HA-v-Myc and pRc-v-Src have been described (34). Transcriptional transactivation analysis using the luciferase reporter system, including the firefly luciferase constructs pGL3-WS5 (pLUC-WS5) and the empty vector pGL3-Basic (pLUC), has been described (33, 34, 36). The eukaryotic expression construct pcDNA3.1-*R*luc used for constitutive renilla luciferase expression, and the empty pcDNA3.1 vector have been described (34). Proliferation of cells treated with curcumin (CRM) was monitored in real time by using the live cell imaging system IncuCyte S3 (Essen Bioscience/Sartorius, Vienna, Austria) as described (33). Cells were seeded in a 24-well dish (Corning, Vienna, Austria), and incubated overnight. Curcumin was then added to final concentrations of 5–40 µM. Cells were monitored for 3 d by phase contrast imaging every 6 h from 16 separate regions per well using a 10× objective.

### Protein Analysis and Antibodies

SDS-PAGE and immunoblotting was carried out as described (34). For co-immunoprecipitation analysis each 3 × 10^6^ cells seeded on four 100-mm dishes were incubated overnight at 37°C and 5% CO_2_ in the absence (two dishes) or the presence (two dishes) of 40 µM curcumin, respectively. Cells were lysed under native conditions in a buffer containing 10 mM sodium phosphate pH 7.2, 150 mM NaCl, 0.5% triton X-100, and 1× HALT™ protease and phosphatase inhibitor cocktail (ThermoFischer Scientific, #48442). The sheared lysate was then clarified by centrifugation, and 1% input samples removed from the supernatants. After addition of the first antibody (5 µl), samples were incubated overnight at 4°C, and then each 25 µl of a magnetic bead protein A/G (Pierce #88802) slurry equilibrated in lysis buffer was added. After a 3-h incubation at 4°C, the beads were pulled down using a magnet, washed 3× with lysis buffer, and once with ultrapure water. The washed pellets were suspended in 15 µl H_2_O followed by the addition of 2× SDS-PAGE sample buffer. After heating at 95°C for 10 min and subsequent centrifugation, each 20 µl of the supernatants were loaded onto a 4–12% Bis-Tris gradient gel as described (37). After SDS-PAGE, the gel was blotted and incubated with the second antibody followed by detection using enhanced chemoluminescence (ECL) as described (37). For densitometry, relative protein levels were determined with ImageQuant TL (GE Healthcare, Vienna, Austria) as described (34).

Specific rabbit antibodies were used recognizing the human MYC (rabbit mcAb #13987, Cell Signaling), human BRAF (mouse mAb #F-7:sc-5284, Santa Cruz), human TRRAP (rabbit pcAb #P2032, Cell Signaling), human EP400 (rabbit pcAb #70301, Abcam), v-Src (mouse mAb #327, Calbiochem), or the hemagglutinin (HA) tag of human influenza virus (mouse mcAb #3808-1, Clontech). The mouse antibody directed against α-tubulin has been described (34).

## Results

### Curcumin Inhibits MYC-Specific Cell Transformation

It has been reported that curcumin has anti-oncogenic properties (26) and therefore we were interested to test if this compound would also influence cell transformation induced by the MYC oncoprotein. The c-*myc* gene (*MYC*) has been originally identified as transduced viral allele termed v-*myc* in the transforming avian acute leukemia virus MC29 (3, 38). To test for oncogenic MYC activity we consequently used an original avian cell system and the retroviral RCAS expression vector (33). The v-*myc* gene fused at its N-terminus with a hemagglutinin (HA) tag was overexpressed in primary quail embryo fibroblast (QEF) and cell transformation monitored in a focus assay, where clonal microtumors result from single transformation events. As a control, the *SRC* oncogene (v-*src*) was tested analogously, which also efficiently transforms avian fibroblasts (34). Increasing amounts of curcumin up to a concentration of 30 µM led to a clear reduction in v-Myc-induced foci, whereas v-Src-induced cell transformation was only slightly affected at a concentration of 30-µM curcumin (**Figure 1A**). Immunoblot analysis, using denaturing SDS polyacrylamide gel electrophoresis showed that the ectopically expressed oncoproteins (HA-v-Myc, v-Src) were efficiently expressed migrating at their expected sizes with apparent molecular weights (*M*_r_) of 53,000 or 60,000, respectively (**Figure 1B**). Surprisingly, extracts from curcumin-treated cells displayed the presence of an additional v-Myc-specific protein with a size significantly larger than the original HA-tagged v-Myc migrating with an apparent *M*_r_ clearly above the 180,000-kDa marker band (**Figure 1B**). Increasing the curcumin concentration up to 40 µM even led to a further reduction in the number of v-Myc-induced foci (**Figure 1C**) accompanied by increasing amounts of the high-molecular MYC-specific complex, and reduced amounts of the ectopic HA-v-Myc protein (**Figure 1D**). This result shows that curcumin efficiently inhibits v-Myc-dependent cell transformation in a specific manner. Moreover, this compound leads to the emergence of a discrete specific immunoreactive protein with a size significantly higher than the 53-kDa ectopic HA-v-Myc, possibly resulting from a curcumin-induced covalent cross-link with another protein, which is resistant to the applied denaturing and reducing SDS polyacrylamide gel electrophoresis conditions.

**Figure 1:** Specific inhibition of v-*myc*-induced cell transformation by curcumin. **(A)** Quail embryo fibroblasts (QEF) were transfected with pRc-HA-v-myc or pRc-v-src encoding the v-*myc* or v-*src* oncogenes, respectively, or with the empty pRc vector as a control using the calcium phosphate method. After the transfection, curcumin was added to the indicated concentrations, and cells were kept under overlay for 16 d. After staining with eosin methylene blue (lower panel), foci were counted on MP12 dishes (n = 2). Vertical bars show standard deviations (SD) from triplicates (upper panel). **(B)** Proteins were analyzed by immunoblotting using equal amounts of cell extracts prepared 2 d after transfection and specific antisera directed against the hemagglutinin (HA) tag of v-Myc, c/v-Src, or α-tubulin (TUBA). **(C)** QEF were transfected and processed as under **(A)** in the presence and absence of curcumin at the indicated concentrations using the pRc-HA-v-*myc* construct (n = 3). Vertical bars show standard deviations (SD) from triplicates (upper right panel). Statistical significance in **(A, C)** was assessed by using a paired Student t‑test (*P < 0.05, **P < 0.01, ***P < 0.005). **(D)** Immunoblot showing HA-v-Myc and α-tubulin expression in cells analyzed in **(C)**. The arrow in **(B, D)** depicts the position of the high-molecular weight protein reacting with the HA antiserum.

### Curcumin Interferes With Transcriptional Activation of MYC

MYC represents a transcriptional regulator of multiple specific target genes both in normal and in neoplastic transformed cells (2, 5). To test if curcumin also affects this central MYC function, a firefly luciferase reporter plasmid (pLUC-WS5) containing the promoter from the MYC-specific target gene *WS5* (33, 39) was transfected into human embryonal kidney cells (HEK293T) representing a suitable cell system to monitor transcriptional promoter activities (35) (**Figure 2**). These cells, which express endogenous MYC at high levels (33) were treated without or with curcumin. Whereas in untreated cells, the *WS5* promoter was efficiently transactivated by the endogenous MYC protein as expected, increasing curcumin concentrations led to a significant reduction in luciferase activities (**Figure 2B**). Immunological analysis of the endogenous 60‑kDa MYC revealed a remarkable gradual reduction of protein levels at high curcumin concentrations (**Figure 2A**). In parallel an augmenting discrete MYC-specific protein band with an apparent molecular weight significantly higher than the band of the 190-kDa marker protein was detected as it has been observed before (cf. **Figure 1**). At a 40-µM curcumin concentration, the endogenous MYC protein band was almost completely replaced by this high molecular weight band, and although these cells express normal α-tubulin levels (**Figure 2A**), a significant arrest in cell proliferation was observed. A decline of MYC-mediated transcriptional activation, and the appearance of a MYC-specific high molecular weight band was also monitored after co-transfection with the renilla luciferase reporter construct pcDNA3.1-RLuc and normalization of firefly *versus* renilla luciferase activities (**Figure 2D**). However, at 40 µM curcumin, both firefly and renilla luciferase activities declined, which may be caused by the observed cell growth arrest, possible triggered by decreased endogenous MYC levels. Nevertheless, the decline of MYC’s transcriptional activation potential at curcumin levels below 40 µM, and the appearance of a MYC-specific high-molecular weight adduct (**Figure 2C**) corroborates our previous observation (cf. **Figure 1**) that curcumin mediates a covalent cross-link of endogenous MYC with a yet unknown protein, thereby impairing its biochemical and biological functions. The result further strongly suggests that the observed decrease in transcriptional activity is due to diminishing levels of the original 60-kDa MYC protein, which could also cause reduced cell proliferation rates that we constantly observed after prolonged curcumin incubation at high concentrations.

**Figure 2:** Inhibition of MYC-dependent transcriptional activation in human embryonic kidney cells (HEK293T) by increasing curcumin concentrations. The firefly luciferase reporter construct pLUC-WS5 specifying the Myc target *WS5* (39) (187.5 ng) was delivered into HEK293T cells (1.5 × 10^5^) *via* lipofection together with 187.5 ng of the empty pcDNA3.1 vector **(A, B)**, or 300 ng pLUC-WS5 with 75 ng of pcDNA3.1-*R*luc specifying the luciferase enzyme from *Renilla reniformis* **(C, D)**. **(A, C)** 6 h after lipofection, curcumin was added at the indicated concentrations, and 30 h after lipofection, protein extracts were prepared. Equal amounts of protein extracts were tested for endogenous MYC expression by immunoblotting using an antibody directed against human MYC. The arrows depict the position the MYC-specific high molecular weight protein. As a loading control, α‑tubulin (TUBA) expression analysis was included. **(B, D)** luciferase activities were measured from cell extracts prepared 30 h after lipofection (n = 2). A 100% activity corresponds to 1.0 × 10^6^ relative light units (RLU) in **(B)**. Firefly and renilla luciferase activities were determined in **(D)** and firefly values normalized using the renilla values as a reference (n = 2). In the applied HEK293T cells, the cotransfection of pcDNA3.1 or pcDNA3.1-Rluc with the empty firefly luciferase reporter pLUC resulted into elevated basal activities, which has not been observed in other cell lines (33, 36). Vertical error bars in **(B, D)** indicate standard deviations (SD) from triplicates. Statistical significance was assessed by using a paired Student t-test (*P < 0.05, **P < 0.01, ***P < 0.005).

### Identification of the 434-kDa TRRAP Protein Covalently Bound to MYC in the Presence of Curcumin

We estimated that the apparent molecular weight of the additional MYC-specific protein is around 500,000 and compared this value with the masses of known proteins interacting with MYC. One of the candidates was the transformation/transcription domain associated protein (TRRAP), a multidomain adaptor protein of the phosphoinositide 3-kinase-related kinases (PIKK) family representing a component of many histone acetyltransferase (HAT) complexes (13). Cell extracts from human embryonic kidney cells cultivated in the presence of 40 µM curcumin were tested by immunoblotting using antibodies directed against MYC and TRRAP (**Figure 3A**). As shown before, curcumin treatment leads to the detection of a MYC-specific protein band with an apparent *M*_r_ of about 500,000. A band of similar size was detected in curcumin-treated cells by using an antibody directed against human TRRAP and migrating slightly above the endogenous 434-kDa TRAPP protein (**Figure 3A**). Quantification of the blots confirmed a significant reduction of endogenous 60-kDa MYC protein levels in the presence of curcumin, and a slight decrease in the level of the endogenous TRRAP, possibly due to the formation of a covalent MYC : TRRAP adduct (**Figure 3A**). To test if the coactivator EP400, which has a similar size as TRRAP and has been found in complexes with MYC (14) is analogously cross-linked with MYC by curcumin, EP400 expression was compared with MYC expression by immunoblotting in the absence and in the presence of curcumin (**Figure 3B**). The analysis showed that under both conditions EP400 migrates slightly faster than TRRAP or MYC : TRRAP and therefore cannot be crosslinked with MYC in the presence of curcumin. Hence, the curcumin-induced covalent cross-link with MYC is specific for TRRAP. To confirm the known physical interaction between MYC and TRRAP *in vivo* (11), two co-immunoprecipitation analyses, both in the absence and in the presence of curcumin were performed (CoIP 1, CoIP 2). Cell extracts were prepared under native conditions from HEK293T cells to preserve the normally occurring non-covalent MYC : TRRAP association in the absence of curcumin, and protein precipitation was performed first with antibodies directed against MYC (CoIP 1), or TRRAP (CoIP 2) (**Figure 3C**). Immunoblot analysis of the precipitates using antibodies directed against TRRAP or MYC, respectively, confirmed that in the tested cells MYC indeed interacts with TRRAP, although the 60-kDa MYC signal in CoIP 2 was rather weak. In the presence of curcumin, as already expected from the result in **Figure 3A**, the curcumin-induced covalent MYC : TRRAP cross-link with a size slightly above the 434-kDa TRRAP protein band could be detected in both co-immunoprecipitations (**Figure 3C**).

**Figure 3:** Identification of the TRRAP coactivator interacting with MYC. **(A)** HEK293T cells were grown for 24 h in the presence of curcumin, and cell extracts prepared and analyzed by immunoblotting. Left panel: besides endogenous MYC with an apparent *M*_r_ = 60,000, a protein band with an apparent *M*_r_ of ~500,000 is detectable under curcumin using a MYC-specific antibody (anti-MYC). Right panel: in the presence of curcumin, the TRRAP-specific antibody (anti-TRAPP) recognizes an additional TRRAP-specific protein migrating above the expected 434-kDa TRRAP protein (arrow). As a loading control, α-tubulin (TUBA) expression was analyzed. Lower panels: relative protein levels of MYC and TRRAP, quantified using the program ImageQuant. **(B)** HEK293T cells were treated with curcumin, and analyzed as under **(A)** using antibodies directed against MYC, TRRAP, EP400, and α-tubulin. The dashed lines in **(A, B)** depict the gel migration position of the MYC : TRRAP adduct migrating above the faint EP400-specific band in the presence of curcumin. The star (*) indicates the position of EP400 degradation products. **(C)** Co-immunoprecipitation analysis using extracts from HEK293T cells treated with or without curcumin and MYC-specific (CoIP 1), or TRRAP-specific (CoIP 2) antibodies (anti-MYC, anti-TRRAP) for the first precipitation under native conditions, and anti-TRRAP (CoIP 1), or anti-MYC (CoIP 2) for the immunological detection after protein blotting, respectively (CoIP 1: due to uneven gel electrophoresis the two input bands migrated slightly faster than the corresponding IP bands). Precipitated proteins were dissociated, and analyzed by SDS-PAGE and immunoblotting using anti-TRRAP or anti-MYC, respectively. As a reference 1% of the lysates were used as input controls. Representative experiments (n = 2) are shown.

### Specificity of the Curcumin-Induced MYC-Specific Cross-Link

Having observed that curcumin not only interferes with basic MYC functions such as cell transformation and transcriptional activation, but also induces a cross-link with TRRAP, we wondered whether these properties were specific for this diarylheptanoid compound, and for the tested oncoprotein MYC (**Figure 4**). For this reason, HEK293T cells were incubated for 24 h with increasing concentrations of curcumin, or the curcumin derivative vanillydene acetone, also termed half-curcumin (**Figure 4G**). As observed in **Figure 2**, increasing curcumin concentrations led to a reduction of endogenous MYC levels and to the emergence of the high-molecular weight MYC : TRRAP protein band (**Figure 4A**), whereas half-curcumin did not show this effect (**Figure 4E**). Consistently, lower amounts of TRRAP were observed at curcumin concentrations above 20 µM, suggesting a TRRAP consumption caused by the TRRAP : MYC cross-link (**Figure 4B**). In contrast, the highly polymeric control protein α-tubulin was not affected by curcumin (**Figure 4D**), and neither down-regulation nor cross-linking were monitored in case of the BRAF oncoprotein representing a dimeric cytoplasmatic protein kinase (**Figure 4F**). For testing a protein different from MYC, and from which it is known that it directly interacts with TRRAP, we selected the tumor suppressor TP53 (18) and analyzed its expression in HEK293T cells under curcumin (**Figure 4C**). This showed that in the presence of increasing curcumin amounts at least one additional TP53-specific protein was detectable migrating with an apparent molecular mass of ~105 kDa. This additional band possibly represents a TP53 dimer suggesting that curcumin also induces cross-links within this tumor suppressor, and thereby could covalently fix a multimeric active structural state. However, no prominent band comparable to the size of the TRRAP : MYC complex was detectable suggesting that the observed cross-link to TRRAP is specific for MYC.

**Figure 4:** Curcumin leads to specific downregulation of the MYC protein thereby inducing a cross-link with TRRAP. **(A–D)** HEK293T cells were incubated with increasing concentrations (5–40 µM) of curcumin. Protein extracts were prepared after 24 h and analyzed by immunoblotting using **(A)** MYC-, **(B)** TRRAP‑, **(C)** TP53, or **(D)** α-tubulin specific antibodies. The arrow in **(C)** depicts the position of a potential cross-linked TP53 dimer. **(E)** HEK293T cells were incubated with increasing concentrations (5–40 µM) of half-curcumin and tested for MYC expression as under **(A)**. **(F)** Expression analysis of the BRAF oncoprotein in the presence or absence of curcumin, or half-curcumin as described under **(A, E)**. **(G)** Structural formulas of curcumin (CRM) and of a non-functional curcumin-derivative termed half-curcumin. A representative experiment (n = 2) is shown **(A–F)**.

### Curcumin Cross-Links MYC Immediately and Arrests Cell Proliferation

Having confirmed the specificity of the curcumin-triggered cross-link between MYC and TRRAP, we were interested in how fast this modification occurs, by monitoring cell proliferation during a time course. For this reason, HEK293T cells were first treated with 40 µM curcumin, and then MYC protein expression was analyzed at different time points of a 2.5-h time period. The immunoblot in **Figure 5A** shows that already 30 min after curcumin addition, the cross-linked MYC : TRRAP complex was detectable suggesting that this chemical modification occurs immediately after intracellular curcumin availability. Furthermore, measuring cell proliferation over a prolonged time period of 72 h showed an immediate decline in the presence of increasing curcumin concentrations (**Figure 5B**) thereby correlating with the time of rapid cross-link formation (**Figure 5A**). Whereas curcumin concentrations of 10–20 µM already diminished the cell proliferation rate, concentrations of 30–40 µM led to a growth arrest, which continued over the entire investigated time period (**Figure 5B**).

**Figure 5:** Immediate formation of the MYC : TRRAP cross-link and inhibition of cell proliferation upon curcumin addition. **(A)** HEK293T cells were incubated with increasing concentrations of curcumin, or the solvent dimethyl sulfoxide (DMSO), and protein extracts prepared after the indicated time points. Proteins were analyzed by immunoblotting using a MYC- or an α-tubulin specific antibody (n = 2). The position of the high-molecular weight MYC protein derivative (p494*^MYC : TRRAP^*) is indicated. **(B)** Proliferation inhibition of HEK293T cells by curcumin. Cells were seeded onto 24-well cell culture plates. The next day, curcumin was added at the indicated final concentrations and cell densities measured every 6 h over a 3-day time period using an Incucyte live cell analysis system. Cells without treatment (DMSO) were used as reference. A representative experiment is shown (n = 2).

### Curcumin Does Not Destabilize the Endogenous TRRAP and MYC Proteins

Incubation of cells with high curcumin concentrations showed that after 24 h the amount of the endogenous 60‑kDa MYC protein starts to gradually decrease, whereas the levels of the MYC-specific high molecular complex (MYC : TRRAP) increase (cf. **Figures 2**, **4A**). This is also accompanied with a loss of MYC functions in terms of transcriptional activation, which could be explained by the lower amounts of the original 60-kDa MYC protein (cf. **Figure 2**). Furthermore, there are decreased levels of TRRAP in the presence of higher curcumin concentrations (cf. **Figures 3A**, **4B**). These declines of MYC and TRRAP in the presence of curcumin could either be caused by increased instability triggered by curcumin, or by sequestration to form the high-molecular TRRAP : MYC adduct. To discriminate between these possibilities, a protein stability test was performed. Curcumin-treated and non-treated HEK293T cells were incubated in the absence and in the presence of the protein translation inhibitor cycloheximide (CHX) (**Figure 6**). A time course of up to 10 h was performed showing that under normal conditions without CHX the MYC and TRRAP protein levels remain stable, whereas in the presence of curcumin MYC and TRRAP levels gradually diminish in favor to formation of the high-molecular MYC : TRRAP adduct (**Figure 6A**). In the presence of CHX, MYC protein levels decrease in non-treated cells as expected due to the short half-time of MYC (33), whereas TRRAP levels remained relatively stable (**Figure 6B**). In curcumin-treated cells, MYC levels only slightly decrease after 2 h but then remain constant (**Figure 6B**). Likewise, the high-molecular MYC : TRRAP derivative in curcumin-treated cells remains stable over the time course. To demonstrate that MYC degradation depends on the ubiquitin/proteasome pathway (40), kinetics were performed in presence of the proteasome inhibitor MG-132 (**Figure 6C**). In both settings, MG-132 led to MYC stabilization confirming previous results (33). Interestingly, the levels of the MYC : TRRAP adduct even increased during CHX and MG-132 treatment (**Figure 6C**). This result shows that curcumin does not shorten the half-times of the MYC or TRRAP proteins, and that the lower levels in curcumin-treated cells possibly result from sequestration to form the MYC : TRRAP adduct, and/or from downregulation of *MYC* mRNA as reported previously (41).

**Figure 6:** Curcumin does not reduce the stabilities of the MYC and TRRAP proteins. **(A)** Equal numbers (2.5 × 10^5^) of HEK293T cells were seeded onto MP24 wells and incubated with increasing concentrations of curcumin or the solvent dimethyl sulfoxide (DMSO), and protein extracts were prepared after the indicated time points. In addition, curcumin- or DMSO-treated cells were incubated in the presence of 25 µM cycloheximide (CHX) **(B)**, or in the presence of CHX (25 µM) plus the proteasome inhibitor MG-132 (5 µM) **(C)**. Protein analysis was performed by immunoblotting using MYC-, TRRAP-, or α-tubulin specific antibodies. The position of the high-molecular weight protein (p494) specifically reacting with the MYC antibody is indicated. A representative experiment (n = 2) is shown. Quantifications of the examined protein expression levels are depicted below each blot.

## Discussion

Numerous attempts have been employed to interfere with the oncogenic functions of the cancer driver MYC in order to obtain tools for efficient treatment of MYC-dependent tumors (42). MYC is a transcription factor belonging to a protein type which is difficult to target by small molecules or peptides due to its particular structure and biochemical function (43, 44). In contrast to oncogenic enzymes, there are no critical surface residues or targetable structures, which are tightly bound by an inhibiting molecule, whereas several drugs against oncogenic kinases exist that are already applied in the clinic or in advanced clinical trials (45). Interfering with signaling pathways upstream of MYC on the transcriptional or post-translational level (42) may represent an alternative, but there is a huge complexity of multiple cross-talking signaling impulses. Comprehensive quantitative descriptions of these pathways by system biology approaches are currently emerging, but so far predictions on how MYC is influenced upon perturbation of a distinct upstream pathway remain difficult. Even when such a pathway is identified, the long and expensive search for inhibitors starts, which realistically takes a decade to end up with a safe compound.

Medicinal plants have a long-standing tradition in the chemotherapeutic treatment of cancer. Multiple plant-derived products have been applied for the treatment of tumors like vinca alkaloids, epipodophyllotoxins, taxanes, or camptothecin derivatives (46). Natural or partially modified compounds from plants may have less undesired side effects and lower the potential toxicity of chemotherapeutic drugs to a certain level. Furthermore, there is still an enormous potential of natural chemicals, which may have chemoprotective efficacies (46). Curcumin as a nutraceutical has been shown to be a safe drug and to be effective against a variety of diseases despite of its low chemical stability, and poor water solubility lowering its bioavailability. Therefore, it has been assumed that not the original curcumin molecule but curcumin degradation or condensation products could be responsible for the various observed biological activities (47). However, as mentioned above the major obstacle in the usage of curcumin is its low bioavailability due to the high hydrophobicity (23). Several attempts to increase the water solubility of curcumin have been done like the development of a water soluble orthogonal self-assembly system using an organoplatinum metallacycle that efficiently delivers curcumin to cancer cells (48). Another possibility is the usage of a biologically active dimethoxy-curcumin, which has a higher metabolic stability than curcumin (49).

The molecular mechanisms how curcumin is effective are not yet clear, although the drug has an impact on the transcriptional regulation of several genes. For instance, curcumin induces transcriptional activation of the tumor-suppressive micro RNA miR-34a, which is paralleled by downregulation of *MYC*, β-catenin, insulin, and *IGFR* mRNAs (41). In addition, the expression of cyclin D1, PCNA, and p21 is modified leading to proliferation inhibition of distinct prostate cancer cell lines (26). Curcumin also inhibits transcriptional activation of the motility, angiogenesis, and metastasis-stimulating factor autotaxin (ENPP2) in human neuroblastomas where the *MYC* gene paralogue *MYCN* is amplified (50). In addition, curcumin downregulates survival mechanisms initiated by the transcription factors NF-κB and AP-1 in prostate cancer cells (49, 51). Another tumor-associated micro-RNA influenced by curcumin is miR-21, which is sorted into exosomes in the presence of this drug, leading to miR-21 depletion in chronic myeloid leukemia cells and upregulation of the tumor suppressor PTEN (52).

Besides, curcumin has anti-inflammatory effects, which could be explained by the induction of the glucocorticoid-induced leucine zipper protein (GILZ). GILZ attenuates inflammation by inhibiting NF-кB and MAP kinase activation (53, 54). Another specific molecular target of curcumin is the dual-specificity tyrosine-regulated kinase 2 (DYRK2), a positive regulator of the 26S proteasome. Structural analysis revealed that curcumin occupies the ATP binding site leading to specific inhibition of the enzymatic activity (55). Consequently, under-phosphorylation of the 26S proteasome leads to impaired proteasome activity and cell proliferation thereby triggering apoptosis in proteasome-addicted breast cancer cells. Furthermore, phosphorylation of the transcription factors MYC and JUN by DYRK2 is required for their degradation in the G_1_/S transition of the cell cycle, an event which is also tumor progression relevant (56). Blocking DYRK2 by curcumin could prevent MYC phosphorylation, which is indispensable for cancer cell growth and consequently inhibit cell transformation. An additional effect of curcumin is the induction of apoptotic pathways thereby inhibiting cell growth and proliferation. Curcumin directly targets a signaling pathway termed spindle assembly checkpoint (SAC), which represents a major cell cycle control mechanism with the E3 ubiquitin ligase APC/C (anaphase promoting complex/cyclosome) as its key regulator. Curcumin binds the APC/C component CDC27 and cross-links its dimeric form thereby inducing programmed cell death, preferentially in cancer cells (57). This interesting property of curcumin to cross-link selected proteins is also relevant in cystic fibrosis, where the compound cross-links cystic fibrosis channel (CFTR) dimers leading to their activation (58).

In this study, we have found that the presence of curcumin interferes with basic MYC functions and induces a cross-link between this oncogenic transcription factor and its coactivator TRRAP. Curcumin efficiently inhibits cell transformation (cf. **Figure 1**) and interferes with transcriptional activation of the cell transformation associated MYC target gene *WS5* (39) (cf. **Figure 2**). In both cases the emergence of a MYC-specific high molecular weight complex was detected in the presence of curcumin, and further analyses revealed that a covalent link between MYC and its transcriptional coactivator TRRAP was established. This is in so far interesting because circular dichroism and nuclear magnetic resonance spectroscopy showed that the interaction of TRRAP with the MYC-Box II induces a structural conformation in an otherwise intrinsically unstructured MYC : TRRAP complex, suggesting that this MYC region is a suitable target to inhibit MYC function (59). Curcumin can form covalent thiol-Michael adducts, which could explain the observed cross-link between MYC and TRRAP complex on a molecular level. The MYC-Box II of human MYC contains one cysteine residue at position 133 and TRRAP has several cysteines in a region, which has been originally identified as MYC-interacting domain (18, 60). It is assumed that sulfhydryl-groups of such cysteine residues form thiol adducts with the curcumin’s enone electrophile of the heptadienone chain (21). Although, we have observed such a cross-link exclusively between MYC and TRRAP (cf. **Figure 4**), this general reaction mechanism could explain the poly-pharmacologic effects of curcumin where the covalent binding to proteins induces functional changes in enzymes, transcription factors like NF-κB (53, 54), or in other proteins (see above).

Human TRRAP represents a highly conserved nuclear protein consisting of 3,859 amino acids with an apparent molecular weight of 434,000 and is a component of several multiprotein complexes such as PCAF, NuA4, BAF53, and TIP60, which display histone acetyltransferase (HAT) activities (11, 61–63). TRRAP is an Ataxia Telangiectasia Mutated (ATM)-related adaptor protein homologous to phosphatidylinositol 3-kinase-related kinases (PIKKs) but without intrinsic kinase activity (11). Thereby, TRRAP acts as an adaptor molecule bridging transcriptional activators with the required HAT function (11, 62), which is required for transcriptional activation and cell transformation triggered by MYC, E2F1, E2F4 proteins (11, 16). However, also tumor suppressors like BRCA1 or TP53 require an interaction with TRRAP for their transcriptional activities (18, 19). In particular the wild type TP53 protein, which binds as a tetramer to diverse DNA targets, is a very efficient cellular defender against neoplastic cell transformation and cancer (64). Covalent cross-linking of TRRAP to MYC could permanently sequester TRRAP with the consequence that the equilibrium of TRRAP binding to its tumor suppressor partners is disturbed (**Figure 7**). Furthermore, in the presence of curcumin there is a drastic reduction in endogenous MYC protein (cf. **Figures 2**, **3A**, **4A**, **6A**), whereas constitutive expression of ectopic v-Myc was almost not affected (cf. **Figure 1**). This could be explained by the fact that normal cells contain much less MYC compared to those expressing this oncoprotein from a viral promoter at very high levels.

**Figure 7:** Schematic diagram showing the proposed mechanism of MYC inhibition by curcumin. **(A)** In proliferating cells or in cells containing aberrantly activated MYC, this transcription factor binds to DNA in complex with the MAX protein and regulates or deregulates the expression of multiple target genes required for cell proliferation or cell transformation. For this activity interaction with other transcriptions factors or coactivators such as TRRAP is required. Likewise, TRRAP also binds to the tumor suppressor TP53 forming functionally active tetramers (64), thereby inducing transcription of the *MDM2* gene, whose protein product then negatively regulates TP53. **(B)** In the presence of curcumin, MYC becomes covalently cross-linked (=) to TRRAP. Thereby, endogenous MYC and TRRAP levels are reduced, whereas TP53 levels remain unchanged mediating the observed growth arrest.

Because the binding sites of MYC and TP53 are juxtaposed in the TRRAP protein (18), it is possible that our observed curcumin-induced MYC cross-link prevents further binding of TRRAP to TP53. The TRRAP : TP53 complex normally activates its transcriptional target *MDM2* representing a proto-oncogene, which encodes an E3 ubiquitin ligase. This enzyme then downregulates wild type TP53 by triggering its proteolytic degradation in the context of a negative feedback regulation (65). Inhibition of *MDM2* transcription due to a lack of TRRAP could result into higher TP53 protein levels which may explain the observed cellular growth arrest (**Figure 7**). Hence, there is a potential synergistic effect of curcumin bifurcating on MYC inhibition and keeping TP53 in its active state.

However, in many tumor cells, TP53 is mutated and possess actually oncogenic attributes (66). In fact, tumors accumulate high levels of mutant TP53, which is also bound and positively regulated by TRRAP suggesting that in cancer cells TRRAP is required to maintain high levels of mutant TP53 (17). Hence, it appears to be reasonable that TRRAP may exert both oncogenic and tumor-suppressive functions depending on whether it interacts with mutant or wild type TP53, respectively. Support for a tumor-suppressive TRRAP function is provided by protein expression analysis in breast cancer tissues revealing that TRRAP expression was significantly lower in breast carcinomas than in corresponding normal breast tissues, and that TRRAP negatively correlates with tumor size but positively with survival time (19). Furthermore, TRRAP is a component of a coactivator complex with HAT activity that is required for the transactivation function of the tumor suppressor BRCA1, which is frequently mutated at the onset of breast and ovarian cancer in women (67).

In summary, the striking finding of a specific covalent cross-link between the two major cellular regulators MYC and TRRAP by the natural food ingredient and industrially used food dye curcumin opens several questions: (1) What is the impact of curcumin on the diverse functions of MYC and TRRAP? (2) How do the altered dynamics between these two proteins influence their impact on other chromatin-remodeling complexes, and (3) what are the consequences for diverse cellular processes such as MYC- or TRRAP-dependent transcriptional programs, DNA repair, or epigenetics? (4) How are diseases, which are negatively influenced by MYC, but abated upon curcumin treatment affected such as cancer, inflammation, neurodegeneration, and osteoporosis? (5) Has this cross-link an activating or an inhibiting effect depending on the multiple pathways in which MYC and TRRAP are implicated? (6) What are the consequences in different cellular contexts, and finally (7) why is curcumin nevertheless such a save drug, despite the potential dramatic consequences as it has been outlined above? In order to address all these questions, comprehensive future studies will heavily dependent on the support by systems biology to cope with the sheer complexity of numerous interdependences between the influenced pathways. Furthermore, the precise determination of the chemical nature and the exact site of the cross-link will enable us to understand the high specificity of this reaction, and elucidate if the cross-linking agent is curcumin itself or a derivative thereof. The respective results will pave the way for medicinal chemistry to adopt this mechanism for the development a possible novel class of drugs.

Nonetheless, the discovery of such a specific molecular mechanism for a plant polyphenol may not be a precedent, as e.g. resveratrol has recently been shown to specifically target the ubiquitin ligase MID1-PP2A complex (68). Both, curcumin and resveratrol are being present in regularly consumed foodstuff, thus raising general epidemiological questions on the impact on public health concerning countries with high consumptions of these substances.

## Data Availability Statement

The raw data supporting the conclusions of this article will be made available by the authors, without undue reservation.

## Author Contributions

RS and MH conceived research. AM, SP, AF, and MH performed experiments and analyzed data. MH and RS wrote the paper. All authors contributed to the article and approved the submitted version.

## Funding

This work was supported by the Austrian Science Fund (FWF) grants FWF-TRP-233-B18 (to RS) and P33662 (to MH).

## Conflict of Interest

The authors declare that the research was conducted in the absence of any commercial or financial relationships that could be construed as a potential conflict of interest.

## Abbreviations

bHLH-Zip, basic helix-loop-helix zipper; CHX, cycloheximide; CMV, cytomegalovirus; Co-IP, co-immunoprecipitation; CRM, curcumin; DMSO, dimethylsulfoxide; ECL, enhanced chemoluminescence; EP400, E1A binding protein p400; HAT, histone acetyltransferase; IB, immunoblot; IP, immunoprecipitation; MBI/MBII, MYC-box I/II; MC29, avian myelocytomatosis virus 29; MDM2, mouse double minute 2 proto-oncogene; MYC, avian myelocytomatosis viral oncogene homolog; PIKK, phosphoinositide 3-kinase-related kinase; QEF, quail embryo fibroblast; RCAS, replication-competent avian retrovirus; SDS-PAGE, sodium dodecylsulfate-polyacrylamide gel electrophoresis; SRC, avian sarcoma (Schmidt-Ruppin A-2) viral oncogene homolog; TP53, tumor protein 53 (p53); TRRAP, transformation/transcription domain associated protein; TUBA, tubulin α.
